This article has been retracted.

# Sinomenine Sensitizes Multidrug-Resistant Colon Cancer Cells (Caco-2) to Doxorubicin by Downregulation of MDR-1 Expression

**DOI:** 10.1371/journal.pone.0098560

**Published:** 2014-06-05

**Authors:** Zhen Liu, Zhi-Jun Duan, Jiu-Yang Chang, Zhi-feng Zhang, Rui Chu, Yu-Ling Li, Ke-Hang Dai, Guang-quan Mo, Qing-Yong Chang

**Affiliations:** 1 Department of Gastroenterology, First Affiliated Hospital of Dalian Medical University, Dalian, Liaoning, China; 2 Department of Neurosurgery, Zhongshan Affiliated Hospital of Dalian University, Dalian, Liaoning, China; University of Navarra, Spain

## Abstract

Chemoresistance in multidrug-resistant (MDR) cells over expressing P-glycoprotein (P-gp) encoded by the MDR1 gene, is a major obstacle to successful chemotherapy for colorectal cancer. Previous studies have indicated that sinomenine can enhance the absorption of various P-gp substrates. In the present study, we investigated the effect of sinomenine on the chemoresistance in colon cancer cells and explored the underlying mechanism. We developed multidrug-resistant Caco-2 (MDR-Caco-2) cells by exposure of Caco-2 cells to increasing concentrations of doxorubicin. We identified overexpression of COX-2 and MDR-1 genes as well as activation of the NF-κB signal pathway in MDR-Caco-2 cells. Importantly, we found that sinomenine enhances the sensitivity of MDR-Caco-2 cells towards doxorubicin by downregulating MDR-1 and COX-2 expression through inhibition of the NF-κB signaling pathway. These findings provide a new potential strategy for the reversal of P-gp-mediated anticancer drug resistance.

## Introduction

Colorectal cancer is one of the most common malignant tumors in gastrointestinal track. In recent years, the incidence of colorectal cancer has significantly increased in china [1]. Surgical resection is the optimal treatment for this kind of cancer, while chemotherapy serves as one of the important adjuvant therapies for its treatment. Currently, the development of multidrug resistance (MDR), a phenotype that cancer cells become resistant to a broad spectrum of chemotherapeutics [2], is a major obstacle in colorectal cancer chemotherapy. It has been shown that emergence of MDR in cancer cells is significantly correlated with the overexpression of membrane pump proteins, including P-glycoprotein (P-gp) [3].

P-gp, encoded by the MDR-1 gene, is a member of the large ATP-binding cassette protein superfamily [4]. P-gp is able to pump a great amount of compounds from intracellular to extra-cellular sites. When cancer cells encounter chemotherapeutic drugs, liposoluble drugs enter cells via the concentration gradient effect. After binding to P-gp, liposoluble drugs are constantly pumped outside of the cell by a process powered by ATP hydrolysis, inducing a continuous decline in intracellular drug levels [5]. Consequently, the drug toxicity on cancer cells is gradually weakened, thereby losing efficacy and, finally, generating drug resistance in cancer cells.

Sinomenine (7,8-didehydro-4-hydroxy-3,7-dimethoxy-17-methylmorphinae-6-one) is one of several alkaloids extracted from the stem of *Sinomenium acutumRehder* & Wilson (Menispermaceae), which has been used traditionally in China and Japan to treat various rheumatic and arthritic diseases [6]. It is worth noting that sinomenine is capable of increasing the absorptive transport of digoxin (a prototypical substrate of p-glycoprotein) and decreasing its secretory transport [7]. Some studies indicate that sinomenine can block activation of NF-Κb [8]. The underlying mechanism of these phenomena remains unclear.

Cyclooxygenase (COX), a rate-limiting enzyme that catalyzes the biosynthesis of prostaglandins (PGs) from the substrate arachidonic acid (AA) and participates in multiple physiological and pathological events. Currently, there are two isoforms of COX: COX-1 and COX-2. In most tissues, COX-1 is expressed constitutively, whereas COX-2 is induced by growth factors, cytokines, and carcinogens [9]. COX-2 is commonly detected in many types of tumor tissues including esophagus, stomach, colon, liver, biliary system, pancreas, breast, lung and bladder cancers [10]. Recent findings have shown that COX-2 expression is positively correlated with P-gp expression in tumor tissue [11]. Relevant studies have demonstrated that COX-2 inhibitors increase the sensitivity of cancer cells to chemotherapeutics by regulating the activity of P-gp [12], [13]. It has been found that celecoxib, a selective COX-2 inhibitor, may downregulate P-gp expression in cancer cells by suppressing the expression of transcription factors such as NF-κB [14], [15]. Several studies indicated that the MDR-1 gene may contain DNA binding sites for transcription factor NF-κB [16], [17].

Some studies indicate that sinomenine inhibits maturation of monocyte-derived dendritic cells through blocking activation of NF-κB [8]. In the current study, we tested the hypothesis that sinomenine may enhance the sensitivity of cancer cells towards antitumor drugs and investigated the potential molecular mechanisms of this effect by directly assessing the effect of COX-2 and NF-κB pathways on P-gp expression.

## Materials and Methods

### Regents and Antibodies

Sinomenine, celecoxib, doxorubicin, 3-(4, 5-dimethyl thiazol-2-yl)-2, 5- diphenyl tetra-zolium bromide (MTT) and dimethyl sulfoxide (DMSO) were purchased from Sigma Chemical Company (St. Louis, MO). Dulbecco’s modified Eagle’s medium (DMEM) and fetal calf serum (FCS) were obtained from GIBCO Life Technology (Grand Island, NY). PGE_2_ and PGE_2_ estimation kit were purchased from Cayman Chemical Co., USA. Triton X-100 was purchased from Amresco, USA. P-glycoprotein (P-gp) mouse anti-human monoclonal antibody, p-IκB-α (Ser 32/36) and IκB-α rabbit anti-human polyclonal antibody were purchased from Santa Cruz Biotechnology (Santa Cruz, CA, U.S.A.). NF-κB p65 rabbit anti-human polyclonal antibody were obtained from Proteintech Group,USA. Monoclonal mouse anti-beta-actin and polyclonal rabbit anti-COX-2 were obtained from Biosynthesis Biotechnology (Beijing, China). FITC labelled goat anti-mouse IgG and FITC labelled goat anti-rabbit IgG were purchased from Amersham Pharmacia Biotech. (Piscataway, NJ).

### Cell Culture

The Caco-2 cell lines employed in this study were purchased from the Chinese Academy of Medical Sciences. Caco-2 cells were cultured in high glucose Dulbecco’s modified eagle’s medium (DMEM, Gibco, Bethesda, MD, USA) culture media containing 10% fetal calf serum at 37°C with 5% CO_2_. MDR-Caco-2 cells were developed by exposure of Caco-2 cells to increasing concentrations of doxorubicin (from 0.1 µM to 1.6 µM in 7 days). Then MDR-Caco-2 cells were incubated without doxorubicin for a week before experiments.

### MTT Colorimetric Assay

The application concentration of sinomenine, celecoxib, PGE_2_ and the capability of sinomenine to sensitize colon cancer cells towards doxorubicin were evaluated using the MTT colorimetric assay. Caco-2 cells and MDR-Caco-2 cells at the logarithmic phase were collected, incubated in a 96-well plate at a concentration of 2×10^4^ cells per well and cultured for 24 h with DMEM supplemented with 10% FCS. Following the attachment of the cells to the wall, DMEM medium (without FCS) containing sinomenine (0, 50, 100, 300, 400, 500, 1000, 2000 µM), celecoxib (0, 5, 10, 15, 20, 25, 30, 35 µM) and PGE_2_ (0, 10^−5^, 10^−4^, 10^−3^, 10^−2^, 10^−1^, 1, 10 µM) were supplemented at a final volume of 200 µL/well for 48 h. After treatment, the medium was removed and the cells were washed twice with DMEM. Then 200 µl DMEM supplemented with 10% FBS and 10% MTT (5 mg/ml) was added. After incubation for another 4 h, the reduced intracellular formazan product was dissolved by replacing 150 µL of DMEM with the same volume of DMSO. The optical density (OD) value was detected at a wavelength of 490 nm with a microplate reader (Bio-rad680, CA, U.S.A.). Four duplicates were designed for each well, and the mean value was calculated three times. The cell growth inhibition rate was calculated from the following formula: cell growth inhibition rate = (1 −OD value in study group/OD value in control group)×100%.

The growth inhibition test was performed to evaluate the capability of sinomenine and celecoxib to sensitize Caco-2 and MDR-Caco-2 cells towards doxorubicin. Following the attachment of the cells to the wall, DMEM medium (without FCS) containing sinomenine (500 µM), celecoxib (25 µM), sinomenine (500 µM) plus PGE_2_ (1 µM) with a interval of 2 h. After incubation for 48 h, the medium was replaced with DMEM (FCS-free) containing doxorubicin (1.6, 2.0, 2.4, 2.8, 3.2, 3.6, 4.0, 5.0, 6.0 µM) for 24 h.

### WST-1 Cell Proliferation Assay

Caco-2 cells and MDR-Caco-2 cells at the logarithmic phase were collected, incubated in a 96-well plate at a concentration of 2×10^4^ cells per well and cultured for 24 h with DMEM supplemented with 10% FCS. Following the attachment of the cells to the wall, DMEM medium (without FCS) containing sinomenine (500 µM), celecoxib (25 µM), sinomenine (500 µM) plus PGE_2_ (1 µM) with a interval of 2 h. After incubation for 48 h, the medium was replaced with DMEM (FCS-free) containing doxorubicin (1.6, 2.0, 2.4, 2.8, 3.2, 3.6, 4.0, 5.0, 6.0 µM) for 24 h. 10 µL of the reagent wst-1 was added (Roche Applied Science, Vilvoorde, Belgium) and incubated for 2 h at 37°C. The optical density was read at 450 nm by microplate reader Labnet (Celbio, Milan, Italy). The wst-1 data were presented as the mean (± S.D.) of triplicate experiments.

### PGE_2_ Estimation

MDR-Caco-2 and Caco-2 cells at a density of 5×10^6^ were seeded in 90 mm culture dishes. They were incubated with or without snomenine (500 µM) for 48 h. At the end of the treatment period, culture medium was collected to determine the amount of PGE_2_ secreted by these cells and stored at)−80°C. The quantitative analysis of PGE_2_ released into the medium was assessed using PGE_2_ immunoassay kit as per manufacturer’s instructions (Cayman Chemical Company, USA).

### Immunocytochemistry

The distribution of P-gp in the cell membrane and nuclear translocation of NF-κB p65 was analyzed by immunocytochemistry as standard procedures. Briefly, Caco-2 and MDR-Caco-2 cells were treated with sinomenine (500 µM) and control medium (without sinomenine) for 48 h and fixed with 4% paraformaldehyde. The cells were incubated with a P-glycoprotein (P-gp) mouse anti-human monoclonal antibody (1∶200 dilution) or a NF-κB p65 rabbit anti-human polyclonal antibody (1∶200 dilution) for 1 h followed by incubation with FITC labelled goat anti-mouse IgG (1∶200 dilution) or FITC-labelled goat anti-rabbit IgG (1∶200 dilution) for 1 h, respectively. Finally, cells were examined under a fluorescence microscope (Carl Zeiss, Thornwood, NY, USA).

### Real-time Relative Quantitative Reverse Transcriptase Polymerase Chain Reaction (PCR) Assay

In order to investigate the effect of sinomenine and celecoxib on P-gp and COX-2 expression, real-time relative quantitative PCR was performed. Cells were plated in 6-well plates with DMEM supplemented with 10% FCS for 24 h. Caco-2 and MDR-Caco-2 cells were treated with sinomenine (500 µM) or celecoxib (25 µM) for 48 h.

Total RNA was isolated with TRIzol reagent (Keygen Biotech Co., Ltd, Nanjing, China), according to the protocol of the manufacturer. The isolated RNA was quantified by spectrophotometry (optical denisty 260/280 nm). The mRNA was then reverse-transcribed into cDNA, according to PrimeScript RT Master Mix Perfect Real Time purchased from Takara Bio Inc. (Dalian, China).

Real-time relative quantitative PCR was performed using the Applied Biosystems 7500 faster Real-Time PCR System with the SYBR Premix Ex Taq (Tli RNaseH Plus) Master Mix purchased from Takara Bio Inc (Dalian, China) in triplicate for each sample and each gene. PCRs were carried out using the oligonucleotide primers listed in Table 1, which describes the size of expected fragments. PCR conditions used were: denaturation at 95°C for 30 s, followed by 40 cycles of denaturation at 95°C for 5 s and 30 s at 60°C for annealing and 30 s at 72°C for elongation. The results were expressed as the ratio value of the CT value for the target mRNA to that of the β-actin mRNA (Ct sample/Ctβ-actin).

**Table 1:** Sequences of the primers used for Real-Time PCR.

Primer name	Primer sequence	Tm(°C)	Expected fragment (bp)
Beta-actin			186
Forward	TGGCACCCAGCACAATGAA	64.7	
Reverse	CTAAGTCATAGTCCG CCTAGAAGCA	62.3	
MDR1			163
Forward	AGGCCAACATACATGCCTTCATC	64.4	
Reverse	GCTGACGTGGCTTCATCCAA	64.6	
COX-2			195
Forward	CTGTAACCAAGATGGATGCAAAGA	62.5	
Reverse	GTCAGTGACAATGAGATGTGGAA	60.0	

### Western Blot Analysis

Western blots were performed based on standard procedures. Briefly, harvested cells were washed twice with cold PBS (pH 7.4). Nuclear extracts were isolated by using the Nuclear/cytosol Fractionation Kit (Keygen Biotech Co., Ltd, Nanjing, China) according to the manufacturer’s recommendations. Total protein were extracted following the manufacturer’s instructions of the test kit from Nanjing KeyGEN Biotech. CO., LTD (China). After determining the protein concentration of samples using bicinchoninic acid (BCA) protein assay, equal amounts of protein samples (30 µg protein) were separated onto SDS-polyacrylamide gels (8% for P-gp, 15% for COX-2, 12% for NF-κB p65, p-IκB-α, IκB-α and beta-actin).

The separated proteins were transferred to a PVDF membrane. After blocking in 5% skim milk in Tris-buffered saline containing 0.05% Tween-20 (TTBS), the PVDF membrane was incubated overnight in blocking buffer with diluted primary antibodies: anti-P-glycoprotein (1∶500 dilution), anti-p-IκB-α (Ser 32/36) and anti- IκB-α (1∶300 dilution), anti-NF-κB p65 (1∶400 dilution), anti-COX-2 (1∶500 dilution) and anti-beta-actin (1∶1000 dilution), at 4°C. Subsequently, the PVDF membrane was washed three times using TTBS, followed by exposure to the secondary antibody: Peroxidase-Conjugated Affinipure Goat Anti-Rabbit and anti-mouse IgG (Biosynthesis Biotechnology, Beijing, China, 1∶2000 dilution). The product bands were photographed, and the density of each product band was quantified by the ChemiDoc XRS documentation system (Bio-Rad Laboratories). The intensity of each signal was corrected using the values obtained from the immunodetection of beta-actin.

### Statistical Analyses

Data are presented as the means ± SE. A preliminary analysis was. carried out to determine whether the datasets accorded with a normal. distribution, and a computation of homogeneity of variance was performed using Bartlett’s test. The means among diverse samples were compared by ANOVA, and multiple comparisons among the groups were conducted using the least-significant difference (LSD) method. If the F values were significant (P<0.05), Dunnett’s method was employed to evaluate individual differences between means, and P<0.05 was considered significant. All of the data were statistically analyzed using the SPSS 11.5 software for windows.

## Results

### Effect of Sinomenine, Celecoxib and PGE_2_ on Caco-2 Viability

Experiments performed by incubating Caco-2 cells up to 48 h with increasing concentrations sinomenine, revealed that this compound does not influence Caco-2 cell viability at concentrations of 500 µM or less (Fig. 1A). A concentration of 500 µM was selected as the application concentration.

**Figure 1:** Cytotoxic effect of sinomenine, celecoxib and PGE_2_ on Caco-2 cells. The cytotoxic effects of indicated compounds on Caco-2 cells were determined by MTT assay. Three independent experiments were conducted. Results are expressed as mean ± SE. Vehicle-treated cells were used as a normalization control. *P<0.5, **P<0.05.

Dose-response and time-course studies demonstrated that celecoxib, a COX-2 specific inhibitor does not affect Caco-2 cell proliferation at doses ranging from 0 to 25 µM (Fig. 1B). Previous studies indicate that celecoxib regulates MDR1 expression by inhibition of COX-2 enzyme activity at a concentration of 25 µM. So, a dose of 25 µM was selected for our experiments [18].

To evaluate whether PGE_2_ could influence the effects of sinomenine, Caco-2 cells were incubated with or without increasing concentrations (0 to 10 µM) of PGE_2_, a COX-2 end product, demonstrated that this compound does not influence Caco-2 cell viability at any concentration tested (Fig. 1C). Studies have shown that PGE_2_ regulates MDR1 expression at a concentration of 1 µM [12], [18], [19], and it is implied that Akt is blocked in the mechanism. Therefore, we chose the dose of 1 µM in our experiments.

### Sinomenine and Celecoxib Enhanced Doxorubicin-induced Ctotoxicity both in Caco-2 and MDR-Caco-2 Cells

To evaluate whether sinomenine and celecoxib might sensitize Caco-2 and MDR-Caco-2 cells to the cytotoxic effects of doxorubicin, Caco-2 and MDR-Caco-2 cells were treated with doxorubicin (10^−5^ to 10 µM) in the absence or presence of sinomenine (500 µM), celecoxib (25 µM), or sinomenine (500 µM) plus PGE_2_ (1 µM) for 48 h. Cell proliferation was determined by MTT assay (Fig. 2 A and B) and WST-1 assay (Fig. 2 C and D). Doxorubicin decreased cell viability dose-dependently both in Caco-2 and MDR-Caco-2 cells with an IC_50_ value of approximately 2.41±0.15 µM and 4.67±0.12 µM (Fig. 2 A), respectively. In MTT assay, cotreatment of Caco-2 cells with sinomenine, or celecoxib, sensitized Caco-2 cells to the cytotoxic effects of doxorubicin with a decrease in IC_50_ values from 2.41±0.15 µM to 1.91±0.16 µM and 1.85±0.2 µM (Fig. 2 A), respectively. Nevertheless, cotreatment with sinomenine plus PGE_2_ had no effect on sensitivity of Caco-2 cells towards doxorubicin.

**Figure 2:** Effects of sinomenine, celecoxib, and sinomenine plus PGE_2_ on cell proliferation in Caco-2 and MDR-Caco-2 cells. Caco-2 and MDR-Caco-2 cells were treated for 48 h with doxorubicin (10^−5^ to 10 µM) alone or in combination with sinomenine (500 µM), celecoxib (25 µM), or sinomenine (500 µM) plus PGE_2_ (1 µM). Cell viability was then determined by MTT assay. Ct group (A and C) refers to doxorubicin-treated Caco-2 group and Ct group (B and D) refer to doxorubicin-treated MDR-Caco-2 group. Data are presented as the mean ± SE. (n = 3) of a representative experiment performed in triplicate. **P<0.01, *P<0.05, compared with doxorubicin-treated Caco-2 group. ##P<0.01, #P<0.05, compared with doxorubicin-treated MDR-Caco-2 group.

Sinomenine and celecoxib also enhanced the cytotoxic action of doxorubicin in MDR-Caco-2 cells, which decreased the IC_50_ value from 4.67±0.12 µM to 2.45 µ±0.14 µM and 2.56 µM±0.11 µM (Fig. 2 B), respectively. Surprisingly, cotreatment with sinomenine plus PGE_2_ had a negative effect on sensitivity of MDR-Caco-2 cells towards doxorubicin with an increased IC_50_ value from 4.67±0.12 µM to 5.35 µ±0.13 µM.

In WST-1 assay, the IC_50_ value of Caco-2 cells decreased from 2.33±0.14 µM to 1.85±0.13 µM and 1.88±0.21 µM (Fig. 2 C). However cotreatment with sinomenine plus PGE_2_ weakened the sensitivity of Caco-2 cells towards doxorubicin with a decrease in IC_50_ values from 2.33±0.14 µM to 2.55±0.17 µM (Fig. 2 C). Sinomenine and celecoxib also enhanced the cytotoxic action of doxorubicin in MDR-Caco-2 cells, which decreased the IC_50_ value from 4.55±0.19 µM to 2.55 µ±0.25 µM and 2.52 µM±0.18 µM (Fig. 2 D), respectively. Amazingly, cotreatment with sinomenine plus PGE_2_ had a negative effect on sensitivity of MDR-Caco-2 cells towards doxorubicin with an increased IC_50_ value from 4.55±0.19 µM to 5.15 µ±0.14 µM (Fig. 2 D).

### Sinomenine Decreased PGE_2_ Release

To examine more closely the involvement of COX-2, the PGE_2_, a COX-2 end product, released from Caco-2 and MDR-Caco-2 cells was determined by ELISA method. The results clearly show a significant increase in the PGE_2_ levels in MDR-Caco-2 cells compared to Caco-2 cells and a significant decline in the levels of PGE2 in MDR-Caco-2 cells treated with sinomenine (Fig. 3).

**Figure 3:** Sinomenine decreased PGE_2_ released from MDR-Caco-2 cells. MDR-Caco-2 and Caco-2 cells were cultured for 48 h in the presence or absence of 500 µM sinomenine, as indicated, and harvested. Supernatants were then collected for PGE_2_ measurement. Data are presented as mean ± SE. (n = 3) of a representative experiment performed in triplicate. Compared to Caco-2 cells, the PGE_2_ levels in MDR-Caco-2 cells significantly increased (P<0.01), which significantly declined in MDR-Caco-2 cells treated with sinomenine (P<0.01).

### Sinomenine and Celecoxib Downregulated the Expression of the P-gp/MDR1 in MDR-Caco-2 Cells

In order to understand the mechanism of resistance developed in MDR-Caco-2 cells, and the mechanism involved in sinomenine and celecoxib sensitizing MDR-Caco-2 cells towards doxorubicin, immunofluorescence cytochemistry, quantitative Real-time PCR, and western blotting were performed. The results showed overexpression of MDR1 mRNA and protein significantly decreased in the presence of sinomenine and celecoxib (Fig. 4).

**Figure 4:** Effect of sinomenine (Sino) on expression of P-gp (MDR1) in MDR-Caco-2 cells. Multidrug-resistant Caco-2 (MDR-Caco-2) cells were developed by exposure of Caco-2 cells to increasing concentrations of doxorubicin (from 0.1 µM to 1.6 µM in 7 days). MDR-Caco-2 cells were incubated without doxorubicin for a week before experiments. Then MDR-Caco-2 cells were treated with or without sinomenine (500 µM) and celecoxib (25 µM) for 48 hours. (**A**) immunocytochemistry targeting P-gp (green). (**B**) Western blot analysis of sinomenine and celecoxib mediated effect on P-gp expression in Caco-2 cells and MDR-Caco-2 cells. Antibody to beta-actin was used to ensure equal loading of protein in each lane. (**C**) The relative band density values in the P-gp expression lanes are described in the bar chat. (**D**) Real-time PCR analysis of MDR1 expression in Caco-2 cells and MDR-Caco-2 cells treated with or without sinomenine. Beta-actin was used as the internal reference for the detection of MDR1 expression. All the results above are expressed as the means ± SE (n = 3) of three independent experiments. *, P<0.05 and **, P<0.01 compared with MDR-Caco-2 group.

### Sinomenine Downregulated the Expression of the COX-2 in MDR-Caco-2 Cells

To understand the role of COX-2 in the development of resistance, and the effect of sinomenine on COX-2 expression, Caco-2 and MDR-Caco-2 cells were treated with or without sinomenine and celecoxib, a COX-2 specific inhibitor, by quantitative Real-time PCR and western blotting. The results revealed that COX-2 is overexpressed in MDR-Caco-2 cells and sinomenine suppressed COX-2 expression (Fig. 5). Besides that, celecoxib has no effect on the expression. We can infer that celecoxib, as a COX-2 specific inhibitor, inhibits the function of COX-2 rather than regulating its expression.

**Figure 5:** COX-2 over expressed in MDR-Caco-2 cells, which could be reversed by sinomenine. MDR-Caco-2 cells were incubated without doxorubicin for a week before experiments. Then MDR-Caco-2 cells were treated with or without sinomenine (500 µM) and celecoxib (25 µM) for 48 hours. (**A**) Western blot analysis of sinomenine and celecoxib mediated effect on COX-2 expression in Caco-2 cells and MDR-Caco-2 cells. Antibody to beta-actin was used to ensure equal loading of protein in each lane. (**B**) The relative band density values in the COX-2 expression lanes are described in the bar chat. (**C**) Real-time PCR analysis of COX-2 expression in Caco-2 cells and MDR-Caco-2 cells treated with or without sinomenine and celecoxib. Beta-actin was used as the internal reference for the detection of COX-2 expression. All the results above are expressed as the means ± SE (n = 3) of three independent experiments. *, P<0.05 and **, P<0.01 compared with MDR-Caco-2 group.

### Sinomenine and Celecoxib Decreased NF-κB Activation

P-gp expression has been clearly correlated to NF-κ B activation [17], [20], [21], which is mediated by the phosphorylation of IκB-α. Subsequently, activated NF-κB p65 subunit translocates to the nucleus and binds to the DNA site, which eventually activates transcription of MDR-1 [22]. To understand the mechanism by which sinomenine and celecoxib enhance the sensitivity of MDR-Caco-2 cells towards doxorubicin, immunofluorescence cytochemistry, quantitative Real-time PCR, and western blotting were performed to detect p65 subunit in nuclear and cytoplasmic p-IκB-α and IκB-α. The results showed that the NF-κB pathway was activated in MDR-Caco-2 cells, while sinomenine and celecoxib suppressed the activation of NF-κB pathway in MDR-Caco-2 cells (Fig. 6).

**Figure 6:** NF-κB pathway was activated in MDR-Caco-2 cells, which was suppressed by sinomenine and celecoxib. Then MDR-Caco-2 cells were treated with or without sinomenine (500 µM) and celecoxib (25 µM) for 48 hours. (**A**) immunocytochemistry targeting P65 (green). (**B**) Western blot analysis of sinomenine and celecoxib mediated effect on nuclear translocation of P65 in Caco-2 cells and MDR-Caco-2 cells. Antibody to beta-actin was used to ensure equal loading of protein in each lane. (**C**) The relative band density values in the nuclear expression P65 lanes are described in the bar chat. (**D**) The relative band density values in the cytoplasmic p-IκB-α lanes are described in the bar chat. All the results above are expressed as the means ± SE (n = 3) of three independent experiments. *, P<0.05 and **, P<0.01 compared with MDR-Caco-2 group.

## Discussion

Chemotherapy serves as one of the important treatments for colorectal cancer. Long-term chemotherapy unavoidably leads to drug resistance and this has become a major challenge to the triumph of chemotherapy. The emergence of drug resistance may correlate with an increase in efflux pump activity, a decrease in drug absorption, the activation of detoxification enzymes, alterations in drug targets and a reduction in cell apoptosis [23]. Previous studies on the efflux pump have shown that P-gp, encoded by the MDR-1 gene, plays an important part, as it pumps drug substance outside to reduce cytotoxicity presented by cancer cells and enhances the resistance of carcinoma to chemotherapeutics. However, the drug resistance presented by cancer cells can be effectively reversed by suppressing P-gp expression and function [24], [25], [26].

Sinomenine, a bioactive alkaloid derived from *Sinomenium acutum*, is used to treat rheumatic and arthritic diseases in China. Sinomenine has a variety of functions including anti-inflammation and immunosuppression [27], [28]. Previous studies have indicated that sinomenine decreased the efflux of prototypical p-gp substrates, such as digoxin and paeoniflorin [6], [7], and sinomenine itself might be a substrate of P-gp [29]. So the regulation methods of sinomenine to P-gp remained unknown. Our results showed that sinomenine downregulated P-gp expression in MDR-Caco-2 cells (Fig. 4) and enhanced the sensitivity of MDR-Caco-2 cells towards doxorubicin (Fig. 2). Some studies have indicated that sinomenine inhibited the expression of COX-2 [30], [31]. Consistent with these results, our findings manifested that sinomenine downregulated COX-2 expression in MDR-caco-2 cells (Fig. 4) and decreased the PGE_2_, an end production of COX-2, released from MDR-Caco-2 cells (Fig. 3).

COX-2, one of the rate-limiting enzyme in the metabolism of arachidonic acid to prostaglandins, is overexpressed in a large number of human primary and metastatic neoplasms [32]. Whether COX-2 is involved in the development of drug resistance characterized by P-gp overexpression is controversial. Many studies showed that COX-2 expression is correlated with P-gp expression [33], [34]. It is reported that adenovirus transfection of COX-2 gene up-regulates MDR-1 gene expression in rat glomerulus cells and maintained the toxicity of adriamycin against renal cells. In the presence of COX-2 inhibitor NS-398, MDR-1 gene expression levels were significantly reduced and the cytotoxicity of adriamycin was enhanced [35]. In line with these findings, we found that the expression of both COX-2 and P-gp are significantly enhanced in MDR-Caco-2 cells. Celecoxib, a COX-2 specific inhibitor, downregulated P-gp expression in MDR-Caco-2 cells and sensitized MDR-Caco-2 cells towards doxorubicin. As stated above, sinomenine inhibited the expression of COX-2 and P-gp. Additionally, when MDR-Caco-2 cells were treated with sinomenine plus PGE_2_, sinomenine failed to enhance the toxicity of doxorubicin towards MDR-Caco-2 cells (Fig. 2).

Previous studies showed that MDR-1 gene contains binding sites for NF-κB, which might correlate with MDR-1 gene expression [16], [17].

NF-κB generally exists as a heterodimer of the p50 and p65 polypeptides, bound in the cytoplasm by the inhibitor protein IκB [36], [37]. Following cellular stimulation by a series of cytokines or pathogens, IκB is phosphorylated by the IκB kinase (IKK) complex at serines 32 and 36, then degraded by the 26S proteosome. Subsequently, NF-κB translocates to the nucleus, where it binds to regulatory elements within the promoter region of target genes. There is evidence that NF-κB was downstream of COX-2 [38], nevertheless, studies have indicated that the down-regulation of COX-2 expression could inhibit NF-κB [39], [40]. In the present study, we found that sinomenine and celecoxib suppressed the activation of NF-κB pathway in MDR-Caco-2 cells (Fig. 6).

In conclusion, we developed a multidrug-resistant Caco-2 (MDR-Caco-2) cell line by exposure of Caco-2 cells to increasing concentrations of doxorubicin, which overexpressed both P-gp and COX-2. Sinomenine downregulated the expression of MDR1 mRNA and protein via NF-κB pathway, and inhibited the expression of COX-2, which was correlated with P-gp expression. Our findings, therefore, provided new insights into the regulation of P-gp expression in multidrug-resistant cells and proposed new potential strategies for the reversal of P-gp-mediated anticancer drug resistance. However, other signaling molecules may also participate in the regulation of the activity of MDR-Caco-2 cells and thus contribute to multidrug-resistant development. Further studies are needed to explore how COX-2, NF-κB and other signaling molecules interact in the development of P-gp-mediated multidrug-resistant in cancer cells.
